The article "Neutrophil-selective deletion of Cxcr2 protects against CNS neurodegeneration in a mouse model of multiple sclerosis" was published in 2020. Journal: J Neuroinflammation.

# Neutrophil-selective deletion of *Cxcr2* protects against CNS neurodegeneration in a mouse model of multiple sclerosis

**DOI:** 10.1186/s12974-020-1730-y

**Published:** 2020-02-04

**Authors:** Yee Ming Khaw, Claire Cunningham, Abigail Tierney, Mayandi Sivaguru, Makoto Inoue

**Affiliations:** 1 Department of Comparative Biosciences, University of Illinois at Urbana-Champaign, Urbana, IL USA; 2 Neuroscience Program, University of Illinois at Urbana-Champaign, Urbana, IL USA; 3 The School of Molecular and Cellular Biology, University of Illinois at Urbana-Champaign, Urbana, IL USA; 4 Carl R. Woese Institute for Genomic Biology, University of Illinois at Urbana-Champaign, Urbana, IL USA

**Keywords:** Multiple sclerosis, CXCR2, Neutrophil, Neuronal cell death, ROS, Dendritic spine loss, CNS

## Abstract

**Background:**

Multiple sclerosis (MS) is a chronic debilitating immune-mediated disease of the central nervous system (CNS) driven by demyelination and gray matter neurodegeneration. We previously reported an experimental autoimmune encephalomyelitis (EAE) MS mouse model with elevated serum CXCL1 that developed severe and prolonged neuron damage. Our findings suggested that CXCR2 signaling may be important in neuronal damage, thus implicating neutrophils, which express CXCR2 in abundance, as a potential cell type involved. The goals of this study were to determine if CXCR2 signaling in neutrophils mediate neuronal damage and to identify potential mechanisms of damage.

**Methods:**

EAE was induced in wild-type control and neutrophil-specific *Cxcr2* knockout (*Cxcr2* cKO) mice by repeated high-dose injections of heat-killed *Mycobacterium tuberculosis* and MOG_35–55_ peptide. Mice were examined daily for motor deficit. Serum CXCL1 level was determined at different time points throughout disease development. Neuronal morphology in Golgi-Cox stained lumbar spinal cord ventral horn was assessed using recently developed confocal reflection super-resolution technique. Immune cells from CNS and lymphoid organs were quantified by flow cytometry. CNS-derived neutrophils were co-cultured with neuronal crest cells and neuronal cell death was measured. Neutrophils isolated from lymphoid organs were examined for expression of reactive oxygen species (ROS) and ROS-related genes. Thioglycolate-activated neutrophils were isolated, treated with recombinant CXCL1, and measured for ROS production.

**Results:**

*Cxcr2* cKO mice had less severe disease symptoms at peak and late phase when compared to control mice with similar levels of CNS-infiltrating neutrophils and other immune cells despite high levels of circulating CXCL1. Additionally, *Cxcr2* cKO mice had significantly reduced CNS neuronal damage in the ventral horn of the spinal cord. Neutrophils isolated from control EAE mice induced vast neuronal cell death in vitro when compared with neutrophils isolated from *Cxcr2* cKO EAE mice. Neutrophils isolated from control EAE mice, but not *Cxcr2* cKO mice, exhibited elevated ROS generation, in addition to heightened *Ncf1* and *Il1b* transcription. Furthermore, recombinant CXCL1 was sufficient to significantly increase neutrophils ROS production.

The article "Neutrophil-selective deletion of Cxcr2 protects against CNS neurodegeneration in a mouse model of multiple sclerosis" was published in 2020. Journal: J Neuroinflammation.

**Conclusions:**

CXCR2 signal in neutrophils is critical in triggering CNS neuronal damage via ROS generation, which leads to prolonged EAE disease. These findings emphasize that CXCR2 signaling in neutrophils may be a viable target for therapeutic intervention against CNS neuronal damage.

## Background

Multiple sclerosis (MS) is a chronic debilitating immune-mediated disease of the central nervous system (CNS) that affects nearly 1 million adults > 18 years of age in the USA [1]. MS symptoms range from common (e.g., pain, spasms, fatigue [2, 3], and muscle weakness [4]) to rarer and more severe (e.g., vision loss [5, 6], physical paralysis, and neurologic disabilities [7, 8]). Immunomodulatory drugs are very effective at shortening the duration of acute flares, decreasing relapse frequencies, and providing symptomatic relief, but there is no cure for MS.

MS has long been considered a white matter disease based on observations of immune-mediated demyelinating lesions in the CNS, but gray matter neurodegeneration is now also appreciated as a major contributor to worsening and permanent disability [9, 10]. Gray matter neuronal pathologies including neuronal apoptosis [11], axonal injury [12], and dendritic spine loss [13] have been observed in the CNS of MS patients. Similarly, gray matter abnormalities have been recapitulated in various animal models of MS, particularly experimental autoimmune encephalomyelitis (EAE) [14], cuprizone toxic demyelination [15], and Theiler’s murine encephalitis virus-mediated demyelination [16] models.

MS disease is believed to be autoimmune in origin, arising when myelin-specific T cells initiate an inflammatory cascade resulting in demyelination and axonal damage [17, 18]. While T cells are recognized as the main driver of MS, elevated numbers of other peripheral leukocytes have been observed in the CNS, suggesting they may also have effector functions in MS. Specifically, a recent report demonstrated that MS patients have a higher circulating neutrophil-to-lymphocyte ratio compared to healthy controls, and the ratio increases with relapse and aggravated disability [19, 20].

Rodent studies have revealed several mechanisms by which neutrophils contribute to disease development. Neutrophils are key regulators of blood-brain barrier permeability, allowing further infiltration of leukocytes into the CNS parenchyma [21, 22]. Neutrophils found in the CNS at the onset of EAE also produce proinflammatory mediators, including TNF-α and IL-1β, which are thought to contribute to the inflammatory cascade within the CNS by stimulating endothelial cell cytokine production and antigen-presenting cell (APC) maturation [23, 24]. Additionally, neutrophils can function as APCs themselves, thereby directly regulating antigen-specific T cell responses [25]. However, their role in neuronal damage has not been rigorously assessed in EAE disease.

The article "Neutrophil-selective deletion of Cxcr2 protects against CNS neurodegeneration in a mouse model of multiple sclerosis" was published in 2020. Journal: J Neuroinflammation.

CXCR2 is thought to be the main receptor in regulating neutrophil chemotaxis [26] and effector function [27] during inflammation. CXCR2 signaling can be activated by receptor ligand CXCL1 which has been shown to be increased in MS patients [28]. Genetic deletion of CXCR2, a chemokine receptor predominantly expressed by neutrophils, prevents development of hindlimb paresis or demyelination in animals subjected to EAE [29] or cuprizone-induced toxic demyelination [30], respectively. The same studies demonstrated that passive transfer of CXCR2-expressing neutrophils to *Cxcr2*^−/−^ mice is sufficient to restore susceptibility to EAE and cuprizone demyelination. Further, we and others have reported that administering a CXCR2 antagonist ameliorates EAE symptoms [31, 32]. In this study, we used neutrophil-specific *Cxcr2* conditional knockout (*Cxcr2* cKO) mice to demonstrate for the first time that CXCR2 signaling in neutrophils is critical for ongoing EAE disease via CNS neuronal damage.

## Methods

### Animals

MRP8Cre (021614) and *Cxcr2*^*fl/fl*^ mice (024638) were purchased from The Jackson Laboratory. MRP8Cre-*Cxcr2*^*fl/fl*^ (*Cxcr2* cKO) mice were bred in our animal facility. Healthy 6–8-week-old male *Cxcr2* cKO and *Cxcr2*^*fl/fl*^ (control wild type) mice were randomly selected and used in this study. All mice were group-housed (2–5 mice per cage) in a specific pathogen-free facility with a 12-h light–dark cycle and were fed regular chow ad libitum. This study was approved by the University of Illinois at Urbana-Champaign Institutional Animal Care and Use Committee (protocol no. 19171).

### EAE induction

To induce EAE disease, complete Freund’s adjuvant, CFA (#F5881, Sigma) containing 400 μg *Mycobacterium tuberculosis*, Mtb (#DF3114-33-8, Fisher), and 100 μg myelin oligodendrocyte glycoprotein _35–55_ peptide (MOG35–55, United Peptides) were subcutaneously administered at 0 and 7 days post-induction (dpi). Pertussis toxin (200 ng/mouse) (#181, List Biological Laboratories, Inc.) was administered on days 0, 2, and 7 dpi. Clinical signs of EAE were scored daily for 40 days in a blinded fashion as follows: 0.5, partial tail limpness; 1, tail limpness; 1.5, reversible impaired righting reflex; 2, impaired righting reflex; 2.5, paralysis of one hindlimb; 3, paralysis of both hindlimbs; 3.5, paralysis of both hindlimbs and one forelimb; 4, hindlimb and forelimb paralysis; and 5, death. We provided water gel and powdered food when the score reached 2 to avoid body weight reduction due to the inability to reach food and water. Disease scoring was performed at midday (during the light cycle).

The article "Neutrophil-selective deletion of Cxcr2 protects against CNS neurodegeneration in a mouse model of multiple sclerosis" was published in 2020. Journal: J Neuroinflammation.

### ELISA measurement of serum CXCL1

Blood was collected via submandibular bleeding from control mice and EAE-induced diseased mice at 9, 21, and 40 dpi. These time points were selected to represent disease onset, disease peak time, and disease late phase, respectively. Serum was isolated and stored at − 80 °C until CXCL1 measurement with a mouse CXCL1/KC Duo set ELISA kit (#DY453, R&D Systems).

### Golgi-Cox neuron staining

At 63 dpi, mice were fixed by 4% paraformaldehyde/PBS infusion, and spinal cords were harvested. Tissue samples were processed using a FD Rapid Stain kit (#NC0292960, FD Neurotechnologies) following the manufacturer’s instructions, embedded in Tissue-tek OCT compound (#23-730-571, Sakura Finetek), and stored at − 80 °C until sectioning. Spinal cords were transversely cut into 50-μm sections using a cryostat (Reichert Jung Cryocut 1800 Cryostat) and mounted onto poly-l-lysine-coated glass slides. After overnight drying, at least 8 sections were developed for Golgi-Cox neuronal staining performed according to the manufacturer’s protocol. After drying, slides were covered with resinous promount and 0.17-μm coverslips.

### Confocal reflection super-resolution (CRSR) acquisition

Samples of Golgi-Cox-stained spinal cords were imaged using a Nikon A1 confocal scanning microscope under the confocal modality and CRSR modality (with minimized pinhole at 0.3 AU) using 20×/0.8 NA objective and 100×/1.49 NA oil objective, respectively [33]. A 405-nm continuous wave laser was used, and the reflectance mirror (BS 20/80) was applied. Images were acquired using 100×/1.49 NA Oil (for dendritic spine analysis) and Plan-Apochromat 20×/0.8 NA (for soma volume analysis) objectives. For dendritic spine analysis, z-stacks of at least 150 intervals were acquired. Pixel dimensions were as follows: x, 0.0628 μm; y, 0.0628 μm; and z, 0.075 μm. Four to eight z-stacks of spinal cord ventral roots from four to eight individual 50-μm-thick spinal cord sections per animal were visualized. A total of 220 dendrites (in 3–4 animals per condition) were included in our analyses (naïve, 60 dendrites; control EAE, 80 dendrites; *Cxcr2* cKO EAE, 80 dendrites) using the filament tracer autopath function (Imaris), as previously described [33, 34]. Importantly, Gaussian filter and background subtraction were applied to z-stacks of cropped individual dendrites prior to tracing filaments. For neuron soma size analysis, neuron soma sizes were determined by individual analysis of soma volumes based on 40-μm z-stacks of Golgi-Cox-stained slices from the ventral horn of the lumbar spinal cord using the Imaris software surface application. Six z-stacks of spinal cord ventral roots from six individual 50-μm-thick spinal cord sections per animal were visualized. A total of 628 neuron somas (in 3–4 animals per condition) were included in our analyses (naïve, 133 neurons; control EAE, 254 neurons; *Cxcr2* cKO EAE, 241 neurons) using the surface rendering function (Imaris).

The article "Neutrophil-selective deletion of Cxcr2 protects against CNS neurodegeneration in a mouse model of multiple sclerosis" was published in 2020. Journal: J Neuroinflammation.

### Mononuclear cell isolation

Brains, spinal cords, spleens, and draining lymph nodes (inguinal and axillary lymph nodes) were harvested from mice at 26–29 dpi. Brains and spinal cords were individually transferred into 5-mL collagenase D (1 mg/mL) (#11088866001, Sigma) solution in 6-in petri dishes, chopped into small pieces using a metal blade, and incubated at 37 °C for 30 min. Tissue slurries were filtered through 70-μm cell strainers. Cells were pelleted by centrifugation at 1500 rpm for 5 min at 4 °C and then suspended in PBS containing 2% FBS. To isolate mononuclear cells from the brains and spinal cords, 70%/30% Percoll gradients were used as previously reported [35]. Spleens and lymph nodes were mashed using frosted glass slides in 5 mL PBS containing 2% FBS, filtered through fine mesh, and pelleted by centrifugation at 1500 rpm/1685 g for 5 min at 4 °C. Cells were washed with hemolysis buffer, pelleted again by centrifugation, and resuspended in PBS containing 2% FBS. Cells were then counted using trypan blue and a hemocytometer.

### Iba1 immunohistochemistry

Spinal cords were harvested from PBS-perfused and 4% paraformaldehyde-fixed mice at chronic disease (33 dpi). Spinal cords were post-fixed in 4% paraformaldehyde overnight and then cryoprotected by immersion in 30% sucrose solution for 24 h. Samples were frozen in OCT compound and stored at − 80 °C until cryostat sectioning. Transverse sections (30 μm) of spinal cords were mounted on poly-l-lysine-coated glass slides. Mounted samples were permeabilized with 0.05% Triton-X for 15 min at room temperature, blocked with 2% BSA for 2 h at room temperature, incubated overnight at 4 °C with goat polyclonal AIF-1/Iba1 primary antibody (#NB100-1028, Novus Biologicals) diluted in PBS, and incubated with chicken anti-goat Alexa 647 secondary antibody (#A21469, Invitrogen) for 2 h. Labeled samples were dried, covered with mounting media (Prolong Gold Antifade Mountant, #P36930, Invitrogen), and sealed with a coverslip. Tissue sections (3 images of ventral roots from individual L4–L6 lumbar spinal cord sections per animal) were visualized using a Nikon A1 confocal scanning microscope at 20× magnification. A total of 2338 Iba1^+^ cells (in 3 animals per condition) were included in our analyses of soma size (control naive, 222 Iba1^+ ^cells; control EAE, 1236 Iba1^+^ cells; *Cxcr2* cKO EAE, 880 Iba1^+^ cells) using the ImageJ *morpholibj* plugin, as previously reported [36].

The article "Neutrophil-selective deletion of Cxcr2 protects against CNS neurodegeneration in a mouse model of multiple sclerosis" was published in 2020. Journal: J Neuroinflammation.

### Flow cytometry

To stain immune cells for flow cytometry, cells were incubated with Fc-Blocker (purified anti-mouse CD16/32 antibody, #101302, Biolegend) in 96-well plates for 7 min and then incubated with fluorochrome-conjugated antibodies for 20 min on ice. Data acquisition was performed on a flow cytometer (Cytek Aurora) and analyzed with Fcs Expression software 6 (De Novo Software). Information from 30,000 gated mononuclear cells was acquired for analysis.

### Neutrophil isolation

Neutrophils from lymphoid organs (spleen and lymph nodes) were isolated by first removing T, B, and DC populations using biotin-labeled anti-CD4 (#100404, Biolegend), anti-CD8 (#100704, Biolegend), anti-CD19 (#115504, Biolegend), and anti-CD11c antibodies (#117304, Biolegend) with streptavidin beads (#19860, Stemcell Technologies), followed by neutrophil positive selection using a biotin-labeled anti-Ly6G antibody (#127604, Biolegend) and dextran-coated magnetic particles (#18556, Stemcell Technologies). Isolated neutrophils were used for reactive oxygen species (ROS) quantitation, co-culture, and qPCR studies.

### Neuronal cell death detection in N2a cells

N2a cells were a gift from Dr. Keith Kelly (UIUC). N2a cells (1 × 10^3^ cells/well) were cultured on cover slips in 24-well plates in 1% FBS/DMEM before initiating co-culture to initiate neuron differentiation [37]. After 3 days, neutrophils were added to N2a neuron culture triplicates at a 2:1 cell ratio and incubated for 18 h at 37 °C with 5% carbon dioxide circulation in a sterile incubator. After 18 h, cells were stained for apoptosis using the FITC Annexin V Apoptosis Detection kit with 7-aad (#640922, Biolegend). Cells were post-fixed in 4% paraformaldehyde. Coverslips were mounted on glass slides with Prolong Gold and stored at 4 °C until image acquisition. A total of 15,007 N2a cells were included in our analyses of 7-aad+ N2a cells (control naïve, 2965 N2a cells examined; control EAE, 4259 N2a cells examined; *Cxcr2* cKO EAE, 7852 N2a cells examined) by manual counting from a blinded experimenter. To evaluate neutrophil-mediated neuronal cell death, value of cell death signal in neuron culture alone was subtracted from that of cell death signal in co-culture of neuron with neutrophil.

The article "Neutrophil-selective deletion of Cxcr2 protects against CNS neurodegeneration in a mouse model of multiple sclerosis" was published in 2020. Journal: J Neuroinflammation.

### Neutrophil ROS detection

Isolated neutrophils were stained with neutrophil markers (Ly6G, CD11b) and a ROS marker in duplicates to detect oxidative stress (CellROX deep red reagent, #C10422, Invitrogen) according to the manufacturer’s protocol. Data acquisition was performed on a flow cytometer (Cytek Aurora) and analyzed with Fcs Expression software 6 (De Novo Software).

### Recombinant CXCL1 treatment to neutrophil in vitro

Wild-type mice were treated with thioglycolate solution (3%, 2 ml/mouse) via i.p. injection. At 24 h after injection, we isolated cells from peritoneal lavage, and isolated neutrophils from them by beads selection, as mentioned above. Then, neutrophils were seeded in a 96-well-plate at 3 × 10^5^ cells/wells. Neutrophils were treated with vehicle (negative control), rCXCL1 (10 or 30 ng/ml, #573702, Biolegend), and LPS (100 ng/ml, positive control, #L4391, Sigma) for 2 h prior to staining with CellROX deep red reagent (Invitrogen). Data acquisition was performed on a flow cytometer (Cytek Aurora) and analyzed with Fcs Expression software 6 (De Novo Software).

### RNA and cDNA preparation for qPCR analyses

Neutrophil total RNA was extracted with an RNeasy Kit (#74106, Qiagen). cDNA synthesis was performed with qScript cDNA SuperMix (#101414-106, VWR). qPCR was performed using KiCqStart SYBR Green qPCR ReadyMix (#250RXN, Sigma Millipore) with an initial denaturing step of 95 °C for 2 min, followed by 40 cycles of denaturation at 94 °C for 3 s and annealing and extension at 60 °C for 30 s. Relative amounts of qPCR triplicates were determined with the *ΔΔCt* method to compare relative expression of target genes and housekeeping genes. Expression of the gene encoding β-actin was used as an internal control.

### Statistical analysis

Statistical analysis was performed using GraphPad Prism 8. All results were evaluated with two-tailed unpaired Student’s *t* tests and *p* values. Data is expressed as mean ± standard error of mean (SEM). A *p* value < 0.05 was considered significant. Animals were randomly used for experiments. All behavior experiments were performed in a blinded fashion. No statistical methods were used to predetermine sample sizes, but our sample sizes are similar to those generally employed in the field [31, 38].

## Results

### Neutrophil-specific *Cxcr2* knockout ameliorates EAE disease

We performed repeated induction of EAE in control wild-type (cont) and neutrophil-specific *Cxcr2* cKO mice, a procedure shown to cause prolonged disease with severe neuronal damage involving CXCR2 [31]. Experimental design is shown in Fig. 1a. Disease onset and severity of motor disturbances were similar in *Cxcr2* cKO mice and control mice at an early disease phase (12–14 dpi) (Fig. 1b). In contrast, Student’s *t* test revealed that control mice showed significantly severe motor disturbances (*p < 0.05) from 15 dpi up to 40 dpi when compared with *Cxcr2* cKO mice that showed weak disease at peak and late phases (Fig. 1b). Repeated induction of EAE induced significant increase in serum CXCL1 levels in EAE-induced mice when compared with non-induced control mice as indicated by data point at 0 dpi (before EAE induction). Notably, at 21 dpi (around peak time), serum levels of CXCR2 ligand CXCL1 were significantly higher than at 9 dpi (onset) and were higher still at 40 dpi in control mice (Fig. 1c). These results suggest that CXCR2 in neutrophils is crucial for EAE disease maintenance and that its function is possibly attributable to highly circulating CXCL1 at peak and late phases.

The article "Neutrophil-selective deletion of Cxcr2 protects against CNS neurodegeneration in a mouse model of multiple sclerosis" was published in 2020. Journal: J Neuroinflammation.

**Fig. 1:** Neutrophil-specific *Cxcr2* knockout ameliorates EAE disease. **a** Schema for experimental design and time schedule. **b** Daily EAE disease scores of wild-type control and neutrophil-specific *Cxcr2* knockout mice (*Cxcr2* cKO), up to 40 days post-induction (dpi). Control EAE, *n* = 10; *Cxcr2* cKO EAE, *n* = 10. **c** Serum CXCL1 levels in control non-induced mice (as indicated by 0 dpi) and EAE-induced mice at 9, 21, and 40 dpi. Note: error bar is present for control group (0 dpi). However, error bar is not visible due to small variation in CXCL1 amount in control groups. Significance was calculated by comparing CXCL1 levels at different time points with 0 dpi. *n* = 8. *p < 0.05, two-tailed unpaired Student’s *t* test

### CXCR2^+^ neutrophils mediate spinal cord neuronal abnormalities at late phase of EAE

We assessed neutrophil *Cxcr2*-dependent morphological changes in Golgi-Cox-stained neurons within the ventral horn of lumbar spinal cord samples in control and *Cxcr2-*cKO mice. At low magnification, we observed gross neuronal anatomical differences between control and *Cxcr2* cKO mice (Fig. 2a). Using our recently developed confocal reflection super-resolution (CRSR) technique [33], Student’s *t* test revealed that control EAE mice exhibited significantly larger (*p < 0.05) neuronal somas than *Cxcr2* cKO EAE mice during late phase disease (Fig. 2b–d). Consistent with abnormalities reflective of neuronal damage and inflammation, neurons from control EAE mice exhibited fewer dendritic spines than control naïve and *Cxcr2* cKO EAE mice (Fig. 2e, f). This suggests that CXCR2 in neutrophils is crucial for CNS pathology during EAE.

The article "Neutrophil-selective deletion of Cxcr2 protects against CNS neurodegeneration in a mouse model of multiple sclerosis" was published in 2020. Journal: J Neuroinflammation.

**Fig. 2:** CXCR2^+^ neutrophils mediate spinal cord neuronal abnormalities. **a** Representative brightfield images of Golgi-Cox staining in the lumbar spinal cord (L4–L6) from control naïve mice, control mice induced with high-dose EAE, and *Cxcr2* cKO mice induced with high-dose EAE. Ventral horn region of interest is identified by red dotted lines. **b** Representative low magnification confocal reflection images of Golgi-Cox stained spinal cord ventral horn. **c** Representative images of volume-rendered neuron soma. **d** Quantitative analysis of neuron soma volume derived from surface rendering of Golgi-Cox-stained neurons, as shown in **c**. A total of 628 neuron somas were included in our analyses (naïve, 133 neurons; control EAE, 254 neurons; *Cxcr2* cKO EAE, 241 neurons) using the surface rendering function (Imaris). **e** Representative raw and rendered CRSR images of Golgi-Cox-stained neuron dendrites. **f** Quantitative analysis of dendritic spine density. A total of 220 dendrites were included in our analyses (naïve, 60 dendrites; control EAE, 80 dendrites; *Cxcr2* cKO EAE, 80 dendrites). Control naïve, *n* = 3; control EAE, *n* = 4; *Cxcr2* cKO EAE, *n* = 4. *p < 0.05, two-tailed unpaired Student’s *t* test

### CXCR2^+^ neutrophils are not required for CNS infiltration of immune cells at late phase of EAE

Student’s *t* tests were performed to reveal that total immune cell counts and counts of various immune cell types in the brain and spinal cord were not significantly different (*p* > 0.05) between control and *Cxcr2* cKO mice at late-phase disease (Fig. 3a, b). We also found no significant differences in immune cell counts in spleens and lymph nodes from control and *Cxcr2* cKO EAE mice (Fig. 3c, d). Thus, the contribution of CXCR2-expressing neutrophils to EAE disease maintenance was not dependent upon neutrophil CXCR2-mediated migration of immune cells into the CNS.

**Fig. 3:** CXCR2^+^ neutrophils are not required for CNS infiltration of immune cells. Numbers of total mononuclear cells, adaptive immune cells (B cells: CD45^+^CD19^+^; CD4^+^T cells: CD45^+^CD3^+^CD4^+^; CD8^+^T cells: CD45^+^CD3^+^CD8^+^), innate immune cells (neutrophils: CD45^+^+Ly6G^high^; dendritic cells: CD45^+^ CD11c^+^; macrophages: CD45^+^CD11b^+^Ly6G^−^CD11c^−^), and CNS resident glia (microglia: CD45^low^CD11b^+^) in the **a** brain and **b** spinal cord of control or *Cxcr2* cKO mice. Numbers of total mononuclear cells, adaptive immune cells (B cells: CD19^+^; CD4^+^T cells: CD3^+^CD4^+^; CD8^+^T cells: CD3^+^CD8^+^), and innate immune cells (neutrophils: CD11b^+^Ly6G^high^; dendritic cells: CD11c^+^; macrophages: CD11b^+^ Ly6G^−^CD11c^−^) in the **c** spleen and **d** lymph nodes of control or *Cxcr2* cKO mice. Control EAE, *n* = 5; *Cxcr2* cKO EAE, *n* = 7. *p < 0.05, two-tailed unpaired Student’s *t* test

The article "Neutrophil-selective deletion of Cxcr2 protects against CNS neurodegeneration in a mouse model of multiple sclerosis" was published in 2020. Journal: J Neuroinflammation.

### CXCR2^+^ neutrophils are not required for microglial activation at the late phase of EAE

We asked if depletion of neutrophil CXCR2 influences microglia activation during EAE. Student’s *t* test was performed to reveal that Iba1^+^ cells in the ventral horn of lumbar spinal cords from control and *Cxcr2* cKO mice at late-phase disease were not significantly different (*p* > 0.05) in soma size (Fig. 4a, b). Thus, neutrophil CXCR2 does not affect microglia activation during EAE, indicating that amelioration of disease severity and spinal cord pathology in *Cxcr2* cKO mice is independent of this process.

**Fig. 4:** CXCR2^+^neutrophils are not required for microglial activation. **a** Representative images of Iba1 immunohistochemistry staining in lumbar spinal cord ventral horns of naïve control, control EAE, and *Cxcr2* cKO EAE mice. Quantitative analysis of Iba1^+^ cell (**b**) soma area as shown in **a**. A total of 2338 Iba1^+^ cells were included in our analyses of soma size (cont naive, 222 Iba1 cells; control EAE, 1236 Iba1^+^ cells; *Cxcr2* cKO EAE, 880 Iba1^+^ cells). Control naïve, *n* = 3; control EAE, *n* = 3; *Cxcr2* cKO EAE, *n* = 3. *p < 0.05, two-tailed unpaired Student’s *t* test

### CXCR2^+^ neutrophils are required for neuronal damage in vitro

We carried out co-culture of neuronal cell line N2a with neutrophils isolated from control and *Cxcr2* cKO mice at late-phase disease. Student’s *t* test revealed that co-cultures with control neutrophils exhibited significantly higher levels of 7-animoactinomycin D (7-aad) (*p < 0.05), a marker of neuronal cell death, than co-cultures with *Cxcr2* cKO neutrophils (Fig. 5a, b), implying neutrophil expression of CXCR2 is necessary to induce neuronal cell death.

**Fig. 5:** CXCR2 in neutrophils is required for neutrophil-induced neuronal damage in vitro. **a** Representative images of N2a neurons co-cultured with neutrophils isolated from control naïve mice, control EAE mice, or *Cxcr2* cKO EAE mice, showing 7-aad neuronal cell death fluorescent signals. **b** Quantification of 7-aad^+^ neurons 18-h post-co-culture with ex vivo neutrophils. A total of 15,007 N2a cells were included in our analyses of 7-aad^+^N2a cells (control naïve, 2965 N2a cells examined; control EAE, 4259 N2a cells examined; *Cxcr2* cKO EAE, 7852 N2a cells examined). *p < 0.05, two-tailed unpaired Student’s *t* test

The article "Neutrophil-selective deletion of Cxcr2 protects against CNS neurodegeneration in a mouse model of multiple sclerosis" was published in 2020. Journal: J Neuroinflammation.

### CXCR2^+^ neutrophils contribute to the proinflammatory phenotype during EAE

We measured ROS, a well-defined trigger of neuronal damage and cell death [39–42]. At late-phase disease, Student’s *t* test revealed that there was a significantly higher percentage of splenic ROS-expressing neutrophils (*p < 0.05) in control EAE samples relative to control naïve mice, control EAE mice, and *Cxcr2* cKO EAE mice (Fig. 6a). To confirm CXCR2 activation signal in neutrophil induces ROS, we isolated thioglycolate-activated neutrophil from naïve WT mice and stimulated with recombinant CXCL1. As expected, CXCL1 treatment increased percentage of ROS-producing neutrophils (Fig. 6b). Further, we measured expression of neutrophil cytosolic factor 1 (*Ncf1*) and myeloperoxidase (*Mpo*), both involved in ROS generation [43], in neutrophils isolated from spleens and lymph nodes of naïve control, control EAE, and *Cxcr2* cKO EAE mice at EAE. Neutrophil treatment of liposaccharide (LPS) was a positive control condition. Consistent with ROS results, neutrophils from control EAE mice exhibited significantly higher expression of *Ncf1* mRNA than neutrophils from control naïve mice (Fig. 6c). However, we observed no differences in *Mpo* mRNA levels (Fig. 6c). Neutrophils from control EAE mice significantly exhibited higher expression *Il1b* than neutrophils from control naïve mice and *Cxcr2* cKO EAE mice. *Tnfa* gene expression levels was not significant different among all three conditions (Fig. 6c). These results demonstrate that CXCR2 in neutrophils is necessary and sufficient for EAE-induced ROS production, revealing a potential mechanism for the observed neuronal damage.

**Fig. 6:** CXCR2 in neutrophils contributes to the proinflammatory phenotype during EAE. **a** Percentage of ROS^+^ neutrophils isolated from spleens and lymph nodes of control naïve mice, control EAE mice, and *Cxcr2* cKO mice. **b** Percentage of ROS^+^ neutrophils isolated from peritoneal space of thioglycolate-injected wild-type mice post-treatment with rCXCL1 at 10 or 30 ng/ml or LPS at 100 ng/ml as positive control. **c** Gene transcription levels of *Ncf*, *Mpo*, *Il1b* and *Tnfa* in neutrophils isolated from spleens and lymph nodes. *p < 0.05, two-tailed unpaired Student’s *t* test

## Discussion

We investigated the role of neutrophil-specific CXCR2 signal in EAE development. Our initial speculation was that CXCR2 signaling in neutrophils is important for initiating disease because neutrophils, which express abundant CXCR2, are early responders during EAE-associated neuroinflammation [23, 44, 45]. However, neutrophil-specific ablation of *Cxcr2* did not suppress early-phase disease development but did affect peak and late phases of EAE. Importantly, we found a large increase in plasma levels of CXCL1, a CXCR2 ligand, during peak and late-phase disease, suggesting that CXCR2 signaling in neutrophils is important at those stages instead of early phase in this neurotoxic EAE model. Because CXCL1 was upregulated in the serum and cerebrospinal fluid of a subset of MS patients [28], CXCR2 signals in neutrophils likely contribute to MS disease.

The article "Neutrophil-selective deletion of Cxcr2 protects against CNS neurodegeneration in a mouse model of multiple sclerosis" was published in 2020. Journal: J Neuroinflammation.

We previously reported that severe CNS neuronal damage and elevated serum CXCL1 [31] are induced during EAE resulting from repeated immunization, the EAE induction method used in this study, hinting that CNS pathology might be affected by neutrophil CXCR2. To test this, we examined the lumbar spinal cord ventral horn because it is the residential address of lower motor neurons and interneurons, both indispensable for normal functioning of hindlimbs [46, 47]. Further, neutrophils are more abundant in the ventral spinal cord than in lateral areas [48]. Neutrophil-specific *Cxcr2* ablation markedly improved spinal cord neuron morphology, as measured by neuron soma size and dendritic density, at late-phase EAE. Changes in neuron sizes are thought to reflect their inflammation state. Increased soma sizes, sometimes also referred to as neuronal swelling [49], have been observed in disease-vulnerable motor neurons during ALS progression [50]. These significant alterations in neuron morphology correlate with the prolonged motor impairments observed in control mice exposed to repeated EAE, which occur up to 40 dpi. Because dendritic spine loss was also reported in MS patients and EAE models [14, 51, 52], we also quantified spine density of dendrites that reside in the ventral horn. Similar to the phenotype of soma enlargement, loss of spines induced by EAE was blunted by neutrophil-specific ablation of *Cxcr2*. Therefore, CXCR2^+^ neutrophils contribute to CNS neuronal damage.

To address the mechanism underlying the role of CXCR2 in neutrophils during EAE, we focused on immune cell infiltration because neutrophils influence migration of other immune cells into the CNS in this model [53, 54]. However, deletion of neutrophil *Cxcr2* did not affect immune cell migration to the CNS. This result is consistent with a previous study demonstrating no deficit in neutrophil recruitment to the CNS in cuprizone-fed mice with global ablation of *Cxcr2* [30]. Additionally, another study demonstrated no change in the number of infiltrating neutrophils to sites of inflammation after administration of a CXCL1 inhibitor [55]. Therefore, CXCR2-mediated neutrophil migration is not implicated in EAE.

Neutrophils are reported to mediate neurotoxic effects by activating CNS resident microglia in cell contact-dependent and cell contact-independent manners [56]. For example, depleting CNS neutrophils significantly decreases in vivo maturation of microglia and infiltrating monocytes, resulting in impaired leukocyte trafficking to the CNS [23] and reduced levels of microglial activation marker CD68 [57]. However, neutrophil-specific loss of *Cxcr2* did not affect microglia activation as evaluated by increases in soma size. Thus, amelioration of spinal cord pathology in *Cxcr2* cKO mice cannot be attributed to changes in microglia effector function.

The article "Neutrophil-selective deletion of Cxcr2 protects against CNS neurodegeneration in a mouse model of multiple sclerosis" was published in 2020. Journal: J Neuroinflammation.

Neutrophils can be direct inducers of neuron damage via enhanced secretion of neurotoxic elastases [58], ROS [59], and extracellular traps [23]. Understanding the range of effector functions that neutrophils can exert upon neurons is important because neutrophils invade CNS parenchyma in multiple contexts of neuroinflammation, including MS, Alzheimer’s disease, and ischemic CNS damage [60]. We found that neutrophils isolated from control EAE mice induced severe neuronal cell death in vitro, and deleting neutrophil *Cxcr2* rescued this effect. Our results suggest that neutrophils may have a direct effect on neuronal damage, and CXCR2 signal is a key regulator of their neurotoxicity.

Neutrophils generate large amounts of ROS, which can trigger neuronal cell death [61]. Exogenous ROS-induced neuronal cell death was shown to be induced via mitochondria-dependent oxidative burst [62]. In this study, deletion of *Cxcr2* in neutrophils suppressed ROS production in neutrophils during EAE. We also found that CXCR2 signal activated by rCXCL1 is sufficient to induce ROS production, which agrees with a previous finding that identified CXCL1 as being a mediator for ROS production in vivo [27]. We also showed that *Ncf1* is upregulated in neutrophils of control EAE mice and suppressed in neutrophils of *Cxcr2* cKO mice. NCF-1 is crucial in the production of ROS [63, 64]. In addition, *Il1b* mRNA is also upregulated in the neutrophil of control EAE mice, but not in *Cxcr2* cKO EAE mice. IL-1β are known to drive direct neuronal damage by activating neuronal apoptosis signaling [65], inducing glutamate excitotoxicity [66]. IL-1β also orchestrates neuron damage by promoting T cell pathogenicity [67, 68] and endothelial cell inflammatory cytokine secretion [69]. Therefore, CXCR2^+^ neutrophil-derived IL-1β may also mediate CNS neuronal damage in EAE. Our study provides evidence of neutrophil-driven neuronal swelling and synaptic loss via CXCR2 signaling which is a key regulator in ROS production.

## Conclusion

Our data provide experimental evidence that neutrophil-specific *Cxcr2* deletion is sufficient to rescue severe disease development and neuronal damage during EAE via preventing ROS generation, implying that neuronal damage results from a CXCR2-mediated ROS generation in neutrophils. We hope that this study will lead to effective therapeutics for preventing CNS neuronal damage in MS patients.

The article "Neutrophil-selective deletion of Cxcr2 protects against CNS neurodegeneration in a mouse model of multiple sclerosis" was published in 2020. Journal: J Neuroinflammation.

## Data Availability

Not applicable.

## Abbreviations

APC: Antigen-presenting cell
cKO: Neutrophil-specific *Cxcr2* knockout
CNS: Central nervous system
CRSR: Confocal reflection super-resolution
EAE: Experimental autoimmune encephalomyelitis
MOG: Myelin oligodendrocyte glycoprotein
MS: Multiple sclerosis
Mtb: *Mycobacterium tuberculosis*
ROS: Reactive oxygen species
